# Effects of Incontro, Alleanza, Responsabilita, Autonomia Intervention Model Combined with Orem Self-Care Model and the Use of Smart Wearable Devices on Perceived Stress and Self-Efficacy in Patients after Total Hip Arthroplasty

**DOI:** 10.1155/2022/5780084

**Published:** 2022-06-09

**Authors:** Mei Cui, Dan Zhao, Hong Wang, Yuqin Zhu, Zhen Wang

**Affiliations:** ^1^School of Nursing, Yangzhou University, Yangzhou, Jiangsu Province 225009, China; ^2^Department of Nursing Administration, People's Hospital of Liuhe District, Nanjing, Jiangsu Province 211500, China; ^3^Medical College of Yangzhou University, Yangzhou, Jiangsu Province 225009, China; ^4^Medical Department, People's Hospital of Liuhe District, Nanjing, Jiangsu Province 211500, China

## Abstract

**Objective:**

To explore the effects of Incontro, Alleanza, Responsabilita, Autonomia (IARA) combined with Orem self-care model and the use of smart wearable devices on perceived stress and self-efficacy in patients after total hip arthroplasty (THA).

**Methods:**

A total of 60 patients after THA in our hospital were enrolled. Patients were randomly divided into control group (IARA intervention model combined with Orem self-care model) and study group (intelligent wearable device combined conference—IARA and Orem self-care model). Harris hip function score, Western Ontario and McMaster Universities Arthritis Index (WOMAC) score, functional independence measure (FIM) score, social support level, perceived stress, and self-efficacy were compared between the two groups.

**Results:**

Harris hip function score, WOMAC score, FIM score, and the level of social support of the study group were higher compared with the control group after operation (*P* < 0.05). Additionally, the perceptual pressure in the study group was lower compared with the control group after intervention (*P* < 0.05). The self-efficacy of the two groups was compared, and the self-efficacy of the study group was higher than that of the control group at 4, 6, 8, and 12 weeks after the intervention, and the difference was statistically significant (*P* < 0.05).

**Conclusion:**

Patients after THA utilize an intelligent wearable device combined with IARA model and Orem self-care model, which can effectively reduce awareness pressure, improve self-efficacy, and facilitate the improvement of the hip fracture.

## 1. Introduction

With the aging of the “baby boomers,” an increasing number of total hip arthroplasty (THA) patients has appeared in recent years in the world [1]. Over the next few decades, the number of THA is predicted to increase [2]. Undoubtedly, this adds to the financial burden and suffering of the patient's life. Studies confirm that patients undergoing total hip arthroplasty (THA) are older and less physically capable [3]. Therefore, early and effective rehabilitation training can avoid joint adhesion, reduce body pain, benefit the recovery of hip joint function, and improve patients' self-care ability [4].

While all postoperative rehabilitation programs should address common strength and range of motion limitations following surgery, every patient's needs should also be taken into account as this group becomes more diverse [5]. Current physical therapy methods following THA address the community as a whole but do not specifically target patients who have higher expectations and wishes for recovery and function. Intervention research on THA is also in the primary stage of exploration, mainly using the Incontro, Alleanza, Responsabilita, Autonomia (IARA). The IARA, which is an Italian acronym, includes two parts namely, the standard procedure and the intervention procedure. Previous study has provided support for the idea that IARA intervention model can be implicated in perceived stress and self-efficacy [6]. By explaining the comprehensive information of THA to patients from shallow to deep, we can gradually deepen their understanding of the interaction between phobia and rehabilitation exercise.

The other nursing theory, called Orem self-care model, was put forward by Dorothea Elizabeth Orem, Master of Nursing Education in the United States [7]. It was gradually applied to clinical practice guidance, education, and research in China in the mid-1980s. It includes self-care theory, self-care defect theory, and nursing system theory [7]. It is widely used in the nursing care of elderly patients undergoing THA. The proposed intervention program based on Orem's self-care model seems to have successfully improved the self-efficacy and reduced the perceived stress of these elderly patients [8, 9]. Recent studies showed that the combination of the IARA and Orem self-care model is also being implemented in clinical trials [10]. These two traditional interventions also have limitations. First, this treatment was not successful in reducing anxiety in healthcare participants, although it did attenuate a non-pathological stressor. In addition, the response rate may have led to the exclusion of perspectives from those who were not appropriately motivated to complete the questionnaire over a long period of time.

In recent years, with the rapid development of wireless technology, cloud computer, and sensor technology, mobile medical wearable devices are becoming a new rehabilitation method for out-of-hospital rehabilitation of patients [11]. Compared with traditional medical services, wearable devices can complete the collection and analysis of patient rehabilitation exercise data to achieve real-time evaluation and helpful guidance [12]. Patients undergoing THA usually have relatively high requirements for life quality due to the need for rehabilitation exercise and self-care abilities.

For this goal, our study designed a scheme of IARA model combined with Orem self-care model and intelligent wearable equipment to test its effectiveness in nursing care of elderly patients with THA.

## 2. Materials and Methods

### 2.1. General Information

From January 2019 to June 2021, 60 patients underwent THA in our hospital. They were randomly divided into the control group and the study group. The control group adopted IARA model combined with Orem self-care model, while the research group adopted the intelligent wearable joint meeting-IARA intervention model and Orem self-care model. In the control group, the age was 45–83 years old, with an average of 60.81 ± 3.63 years, including 18 males and 12 females, 18 cases of the left hip and 12 cases of the right hip, whereas in the study group, the age was 44–85 years old, with an average of 60.96 ± 3.82 years. There were 16 males and 14 females, and the injured sites were the left hip (*n* = 15) and the right hip (*n* = 15). There was no statistical significance in the general data of the two groups. This study was approved by the Medical Ethics Association of our hospital, and all patients signed informed consent.

Inclusion criteria are: (1) the function of the hip joint is limited due to various reasons, which brings great inconvenience to the patient's life, and the patient has decided to perform hip arthroplasty for treatment; (2) the patient can independently complete the questionnaire survey and scale evaluation; (3) willing to participate and sign the informed consent form and the compliance is good; (4) there is no serious dysfunction of important organs such as heart, brain, lung, and kidney; (5) no disturbance of intelligence and consciousness; (6) unilateral hip joint patients, age ≥18 years old, ≤90 years old; and (7) metal-on-polyethylene (M-on-PE) was used in THA.

Exclusion criteria are: (1) those who are unwilling to participate in this experiment; (2) patients who are unable to complete the questionnaire and scale evaluation due to language, cognitive, and other reasons; (3) active infection in any other part of the body; (4) patients with mental retardation, unclear consciousness, major organ dysfunction or malignant tumors; (5) diseases that significantly increase the incidence of sequelae or mortality; and (6) neuroarthropathy, lower limb myodynamia or relative insufficiency and rapidly progressive neurological diseases.

### 2.2. Treatment Methods

The control group received IARA intervention model combined with Orem self-care model. Before the study, a research group was set up with the consent of the leaders of the relevant departments. The team members include two orthopedic doctors, one psychological counselor, one rehabilitation physician, four orthopedic nurses, two rehabilitation nurses, and three nursing managers. Among them, there are four senior titles and six intermediate titles. We should record the basic data of the patients, improve the preoperative orthopedic examinations, be familiar with the patients' medical records, and choose the communication methods suitable for the patients according to their educational level. For example, patients with a lower level of education can communicate in intuitive forms such as dialects, pictures, and metaphors, whereas those with a higher level of education can explain some easy-to-understand professional knowledge. Step-by-step diagram of the IARA training and Orem self-care model nursing sessions were shown in Tables 1 and 2.

The research group uses the smart wearable joint meeting-IARA intervention model and Orem self-care model. IARA intervention model and Orem self-care model are the same as the control group. Smart wearable devices are used as follows: the Smart + connected wearable device used in the study to measure and record the range of motion of the joint. The device consists of a wearable intelligent bandage (built-in attitude sensor), medical terminal Mini Program (bone care terminal: menu bar includes patients, plan templates, team management, popular science articles, and consultation settings), and patient side APP (bone know: menu bar includes training, discovery, doctor, and patient management). Patients connect the wearable bandage to GushiTong APP through Bluetooth, then fix the bandage in the correct position according to the guidance of the APP training module, and carry out rehabilitation training according to the individual rehabilitation plan pushed by medical care (different stages of the rehabilitation program are preset in the system). The built-in sensor of this device can record the angle, frequency, and training time of the patient's rehabilitation action in real-time, and the system can automatically judge whether the patient's rehabilitation exercise is up to the standard or not through the preset times and angles. The software will give a warning when it exceeds or does not reach the set value. Patients can record rehabilitation data only after completing the preset minimum number of effective times. Through the feedback of objective data, the medical and nursing side can evaluate, analyze, and adjust the rehabilitation plan in real-time, and carry out long-distance and fine management after the operation. On the other hand, patients can understand their own rehabilitation status directly through the data and obtain rehabilitation-related knowledge. Concomitantly, this device has a reminder function to urge patients to carry out rehabilitation training by sending text messages every day.

### 2.3. Observation Index

#### 2.3.1. Harris Hip Joint Function Score

Harris hip joint function score scale [10]: the efficacy of hip disease was evaluated by medical staff. The scoring system included 4 dimensions of pain, function, deformity, and range of motion, with a total of 10 items and a total score of 100 points. The higher the score, the better the hip function.

#### 2.3.2. Western Ontario and McMaster Universities Arthritis Index (WOMAC) Scoring

Western Ontario and McMaster University Arthritis Index (WOMAC) [11] reflects the severity of the joint injury and the recovery of joint function according to symptoms and signs, tend to be self-assessed by patients and pay more attention to their subjective experiences including pain, stiffness, joint function in three dimensions, a total of 24 items, a total score of 96, the higher the score, the more serious the joint damage.

#### 2.3.3. FIM Scoring

The functional independence measure (FIM) [12] was used to evaluate the patients including self-care ability, sphincter control, transfer, actionability, communication, and social cognition five dimensions, a total of 18 items, a total score of 18–126, the higher the score, the better the functional independence of the patient. The FIM scale has good intra-and inter-group reliability and good internal consistency.

#### 2.3.4. Social Support Level

Evaluation of social support level [11]: social support rating scale was used to measure the objective support dimension, subjective support dimension, and support utilization dimension. There are 10 items, and the corresponding items in three dimensions are 3 items (2, 6, 7 items), 4 items (1, 3, 4, 5 items), and 3 items (8, 9, 10 items). Among them, items 1–4 and 8–10 all adopt 1–4 Likert 4 score. Other items are scored according to the selection, the higher the score, the higher the level of social support, 22 points are the critical value [7, 8].

#### 2.3.5. Perceptual Stress Scale

The Chinese version of Perceptual stress scale (CPSS): it was compiled by American scholar Cohen in 1983 [12]. The scale mainly measures the stress perception of individuals. The scale consists of 14 items that are assigned into two dimensions: tension and out of control. Using the Likert 0–4 score and the 5-grade score, the total score was 56. The higher the score, the greater the pressure perceived by the patients, including 0–28 as normal pressure level, 29–42 as high-stress level, and 43–56 as excessive stress level. In this study, the Cronbach's *α* coefficient of the scale was 0.781.

#### 2.3.6. Self-Efficacy

Rehabilitation exercise self-efficacy evaluation [13]: rehabilitation exercise self-efficacy scale (SER) was enrolled for evaluation. The scale included physical exercise self-efficacy and coping self-efficacy, with a total of 12 items. The items were scored by Likert 11 grade, including “unable at all” to “without any difficulty,” with a score of 0–10 points and a total score of 0–120 points [4, 5].

### 2.4. Statistical Analysis

The data were sorted out and statistically analyzed by IBMSPSS20.0 software, the measurement data were described by mean ± standard deviation $\bar{x}\pm s$, repeated measurement analysis of variance or *t*-test were used for inter-group and intra-group comparison, and *χ*^2^ test was used for inter-group comparison. The difference was statistically significant when *P*-value was less than 0.05.

## 3. Results

### 3.1. Comparison of Harris Hip Joint Function Score

Harris hip function score was compared. Before nursing, there was no significant difference (*P* > 0.05). After nursing, the Harris hip function score of the two groups was improved. In addition, the Harris hip function scores at 4, 6, 8, and 12 weeks after operation in the study group were higher than those in the control group, and the differences were statistically significant (*P* < 0.05). All the results are indicated in Figure 1.

### 3.2. WOMAC Score Comparison

We compared the WOMAC scores of the two groups. Before nursing, there was no significant difference (*P* > 0.05), wheras after nursing, the WOMAC score of the study group was lower compared with the control group at 4, 6, 8, and 12 weeks after operation, and the difference was statistically significant (*P* < 0.05). All the results are indicated in Figure 2.

### 3.3. FIM Score Comparison

Then, we compared the FIM scores of the two groups. Before nursing, there was no significant difference (*P* > 0.05); wheras after nursing, the FIM score of the study group was higher compared with the control group at 4, 6, 8, and 12 weeks after operation, and the difference was statistically significant (*P* < 0.05). All the results are indicated in Table 3.

### 3.4. Comparison of the Level of Social Support

The level of social support was compared. Before nursing, there was no significant difference (*P* > 0.05). After nursing, the level of social support at 4, 6, 8, and 12 weeks after surgery in the study group was higher compared with the control group, and the difference was statistically significant (*P* < 0.05). All the results are indicated in Table 4.

### 3.5. Perceived Stress Comparison

The perceived stress between the two groups was compared. Before nursing, there was no significant difference between the two groups (*P* > 0.05); whereas after nursing, the perceptual pressure decreased in both groups, and the difference was statistically significant (*P* < 0.05). The perceptual pressure in the study group was lower compared with the control group at 4, 6, 8, and 12 weeks after surgery, and the difference was statistically significant (*P* < 0.05). All the results are indicated in Table 5.

### 3.6. Comparison of Self-Efficacy

The self-efficacy of the two groups was compared. Before nursing, there was no significant difference between the two groups (*P* > 0.05); whereas after nursing, the self-efficacy of the two groups increased. The self-efficacy of the study group at 4, 6, 8, and 12 weeks after operation was higher compared with the control group, and the difference was statistically significant (*P* < 0.05). All the results are indicated in Table 6.

## 4. Discussion

THA is one of orthopedic surgery's most cost-effective and consistently successful procedures [13]. It provides consistent results for people with advanced degenerative hip osteoarthritis, such as pain reduction, restoration of function, and improved quality of life. After THA, the physical therapy and the mental intervention measures are required by patients. Either way, the patients usually benefit from these no-drug therapies to help patients regain their normal function. Outpatient intervention therapy is the final step before returning to full function after a total hip replacement [14].

Therefore, how to rebuild functional rehabilitation and the prevention of various complications has become an important topic in clinical scientific research. The Harris hip function score of the patients in our study was improved after the nursing of IARA and Orem self-care model intervention. Furthermore, the Harris hip function score of the patients with smart wearable devices was higher compared with those without smart wearable devices. Our results are consistent with the previous report [15]. Our study again provides positive clinical evidence to support this notion. Patients can access rehabilitation resources anytime and anywhere without the constraints of time and space. Alexander et al. constructed a network physical system named Rehab Tracker [16]. Rehab Tracker can combine communication devices and medical equipment, providing patients with auxiliary electrophysical rehabilitation and recording doctor-patient conversation data. In addition, our data have shown that FIM score and WOMAC score were higher compared with those without smart wearable devices during nursing. A combination of smart wearable devices, IARA, and Orem self-care model is capable of improving postoperative hip function in THA patients. Our study has suggested a promising future for smart wearable devices combined with clinical care to improve patient prognosis.

After nursing, the level of social support in the study group was higher compared with the control group. Social support refers to the psychological and material resources provided by a social network to help individuals cope with stress [17]. The results of our trial are consistent with previous reports.

The researchers have pointed out that the mobile medical system still needs to be further improved [17]. Many clinical trials have proved that emotion regulation is one of the key factors in IARA intervention, which can relieve patients' stress and reduce their postoperative fear of movement [18]. Previous studies have shown that patients who participated in IARA training had positive mood regulation, anxiety, and stress scores 6 months after the end of the intervention [6]. Furthermore, a positive relationship has been observed between emotion regulation, perceived stress, and anxiety [6]. Some scholars believe that, in the intervention of IARA, the first meeting is disease education; the second meeting is to use a “breathing bottle” to systematically explain the respiratory system; and the third meeting is to release patients' potential through self-efficacy and reestablish a balanced state of health [19].

Nurses help patients complete self-care activities and make up for the deficiency of patients' self-care [18]. According to the supportive education system, older patients receiving THA must learn and be able to self-care, and patients must be able to complete self-care activities. Nurses assist patients by providing psychological support, technical guidance, and a safe atmosphere. In the meantime, it has reinforced the nurse-patient relationship, increased job satisfaction, improved communication and understanding between the nurse and the patient, and supported the nurse-patient relationship's harmonic development [20].

A large number of studies have pointed that outpatient-based rehabilitation is easily limited by time, distance, and cost [21, 22]. As a new approach to telemedicine, wearable devices can quantify the exercise behavior of different patient groups. Quantitative and continuous real-time information feedback can effectively make up for the current shortcomings of out-of-hospital rehabilitation. A qualitative study by Sharma et al. interviewed 10 orthopedic rehabilitation professionals in a semi-structured interview [23], which showed that clinicians believed that wearable technology could be employed as a medium to track the measured data in real-time, which had great potential in assisting the rehabilitation process. A British survey on the acceptance of remote rehabilitation tools by patients after THA showed that most patients had high acceptance of remote rehabilitation and it was able to improve the ability of self-management, with the effect of improving exercise intervention significant [24]. According to the results of the study, digital intervention technology and physiotherapy are integrated to create a personalized rehabilitation plan for THA patients. This study found that patients were not limited by time and space, and could obtain rehabilitation resources anytime, anywhere. The researchers also pointed out that the mobile medical system still needs to be further improved. Tang Tang attempted to merge wearable technology with gaming components to investigate the feasibility and effectiveness of intelligent wearable equipment with joint measurement, feedback, and neuromuscular electrotherapy in-home rehabilitation of THA patients [25]. Some scholars analyzed that the cost-effective wearable sensor could objectively quantify the clinical movement of the population [26–29]. However, further clinical empirical investigations in the field of sports injury are needed to validate its accuracy and availability.

## 5. Conclusion

The smart wearable device combined with IARA model and Orem self-care model can effectively reduce the conscious pressure of patients after THA, improve self-efficacy, and promote recovery after THA. Therefore, it is advised that this nursing program be considered as part of the treatment strategies for these patients.

## 6. Limitation

Some limitations of this study should be addressed when interpreting the results and planning future research. To begin, the sample size was modest (60 cases were included). No multicenter studies were carried out. Second, the patients included in our study were selected, mainly to avoid comorbidities or post-surgery complications. This may limit the generalizability of the results. In the future, it is mandatory that multicenter clinical trials with large sample size should be performed.

## Figures and Tables

**Figure 1:** Comparison of Harris hip function Score.

**Figure 2:** Comparison of WOMAC scores between the two groups.

**Table 1:** The IARA training sessions are depicted in a step-by-step diagram.

	Content of the meeting
First intervention	The nurse hands out the THA rehabilitation Education Manual, asks the patient to read the contents, discusses with the patient and family to establish rehabilitation goals according to the plan, taking into account the patient's fear of movement and cognitive ability; the intervention time is from admission to operation
Second intervention	The nurse communicated with the patients about postoperative exercise plans, precautions for the use of prosthesis. and precautions for the use of double crutches; the rehabilitation nurses educate about phobias, explain the mechanisms by which phobias affect rehabilitation exercises, and emphasize the benefits of early exercise; the orthopedic surgeons pay attention to their fears during the communication process, answer questions, and meet the appropriate needs in a timely manner; the intervention lasted from the second to the fourth day postoperatively
Third intervention	To further improve the long-term plan, the rehabilitation nurse checked and guided the patient's rehabilitation movements, emphasizing body balance and proprioceptive training to avoid secondary hip injuries caused by human factors such as falls; the nursing staff reminded the patient to return to the hospital for regular review and to consult via WeChat and telephone if there was any doubt; the intervention lasted from the fifth day after surgery to discharge.

**Table 2:** The Orem self-care model of nursing is depicted in a step-by-step diagram.

	Content of the nursing
Complete compensation nursing	THA patients who were not fully awake after anesthesia and who were unable to take care of themselves should use a full compensatory care system to compensate for the patient's ability to take care of themselves with medical support; the intervention time is on the first day after surgery
Partial compensatory nursing	When the patient's vital signs are stable and conscious, the nurse should disseminate knowledge of postoperative rehabilitation exercises and give partial compensatory care; mobilize the patient's initiative and improve their self-care ability and behaviors, with emphasis on assistance, guidance, and education; the intervention time lasted from the second day to the first week after surgery
Support education and nursing	Nurses use the support education system to provide psychological support, counseling, health education, and nursing guidance to patients; the nurse provides information and health education to the patient and their family so that they can actively participate in the care activities, thus achieving a speedy return to independent living; the intervention lasted from the first week after surgery to discharge

**Table 3:** Comparison of FIM scores between the two groups ($\bar{x}\pm s$, Points).

Group	*N*			Before nursing	4 weeks after surgery	6 weeks after surgery		8 weeks after surgery	12 weeks after surgery
C Group		30	97.86 ± 9.56		103.82 ± 5.45	108.84 ± 5.97	110.72 ± 6.84		180.74 ± 4.29	
R Group		30	97.94 ± 9.46		115.93 ± 4.96	119.87 ± 3.86	123.83 ± 4.66		125.75 ± 5.64	
*t*			0.032		9.000	8.497	8.675		42.504	
*P*			0.974		<0.01	<0.01	<0.01		<0.01	

**Table 4:** Comparison of social support level between the two groups ($\bar{x}\pm s$, Points).

Group	*N*	Before nursing	4 weeks after surgery	6 weeks after surgery	8 weeks after surgery	12 weeks after surgery
C Group	30	10.28 ± 3.55	11.83 ± 1.45	12.94 ± 3.31	15.85 ± 3.55	19.72 ± 2.15
R Group	30	10.27 ± 3.41	13.84 ± 3.84	15.74 ± 3.45	17.84 ± 3.81	21.84 ± 1.44
*T*		0.011	2.682	3.207	2.093	4.487
*P*		0.991	<0.01	<0.01	0.040	<0.01

**Table 5:** Comparison of perceived stress between the two groups ($\bar{x}\pm s$, Points).

Group	*N*	Before nursing	4 weeks after surgery	6 weeks after surgery	8 weeks after surgery	12 weeks after surgery
C Group	30	38.83 ± 2.45	34.69 ± 3.44	30.81 ± 4.23	25.83 ± 3.41	21.85 ± 3.81
R Group	30	38.91 ± 2.45	30.85 ± 2.24	25.86 ± 4.33	21.44 ± 3.53	15.68 ± 4.31
*T*		0.126	5.123	4.478	4.899	5.874
*P*		0.899	<0.01	<0.01	<0.01	<0.01

**Table 6:** Comparison of self-efficacy between the two groups ($\bar{x}\pm s$, points).

Group	*N*	Before nursing	4 weeks after surgery	6 weeks after surgery	8 weeks after surgery	12 weeks after surgery
C Group	30	56.94 ± 4.91	60.94 ± 4.31	65.48 ± 5.42	70.84 ± 5.42	75.97 ± 4.23
R Group	30	56.83 ± 4.83	65.24 ± 4.91	71.65 ± 4.33	78.85 ± 4.23	85.95 ± 4.19
*t*		0.087	3.604	4.871	6.381	9.180
*P*		0.930	<0.01	<0.01	<0.01	<0.01

## Data Availability

No data were used to support this study.
